# The Application Trend of Digital Finance and Technological Innovation in the Development of Green Economy

**DOI:** 10.1155/2022/1064558

**Published:** 2022-07-12

**Authors:** Ya Zhou

**Affiliations:** School of Marxism, Southeast University, Nanjing, Jiangsu 211189, China

## Abstract

Based on the perspective of digital finance and technological innovation, this paper analyzes its application in economic development, green economy, and sustainable development. With the continuous development of technological economy, methods such as artificial intelligence, Internet of Things, big data, and cloud computing become increasingly mature. Economic development is inseparable from the empowerment of technology. In this paper, firstly, we introduce the basic concepts and main forms of digital finance and technological economy and list the cutting-edge technologies including blockchain, VR, sharing economy, and other modes. Then, we analyze the application trend of technology economy. Finally, we analyze the examples of digital finance and technological innovation in detail, including tourism economy, digital marketing, sharing economy, smart city, digital healthcare, and personalized education, three hot topics of technology intersection and integration. In the end, we put forward prospects for the development of a digital economy, digital finance, and technological innovation.

## 1. Introduction

In 2020, the added value of the digital economy in 47 countries reached US $32.6 trillion, up by 3.0 percent year-on-year in nominal terms and accounting for 43.7 percent of the GDP. The digital economy in developed countries is large in scale and accounts for a high proportion. In 2020, the digital economy reached US $24.4 trillion, up by 3.0 percent year-on-year and accounting for 54.3 percent of the GDP. The digital economy in developing countries is smaller at $8.23 trillion and growing faster, reaching 3.1 percent in 2020. The US continued to be the world's largest digital economy, with a size of US $13.6 trillion in 2020, while China ranked second with a size of US $5.4 trillion. Germany, Japan, and the UK ranked third through fifth with $2.54 trillion, $2.48 trillion, and $1.79 trillion, respectively. In the development of the digital economy, developed countries have advantages over developing countries.

As early as 1912, Schumpeter made a preliminary study on the relationship between financial development and technological innovation [1]. However, it was not until the promotion of financial marketization and the development of the third scientific and technological revolution that the study of the relationship between financial development and technological innovation formally attracted the attention of scholars at home and abroad and became a hot topic of academic debate [2, 3]. With the development of physical finance and the arrival of the third wave of scientific and technological revolution, finance in a new form of digital valuation is active in the public vision. In a short period of more than 10 years, digital finance research is in the ascendant. At present, technology-innovative enterprises are facing serious financing constraints, which can be roughly attributed to the following reasons. First of all, technology-innovative projects are characterized by long investment cycles, large capital input, high risk, high transaction cost in traditional financial markets, overall planning mode of capital-lending projects, and cumbersome review process, which may lead to the enterprise's innovation projects missing the best research and development period due to the fracture of the capital chain. Secondly, the information asymmetry between money supply and demand restricts the external channels of enterprise development and financing. Traditional financial intermediaries cannot participate in innovative projects, nor can they prevent moral hazard problems that enterprises may face by establishing an effective mechanism of money supply pre review, event tracking and post supervision [4]. Finally, the poor quality of enterprise credit guarantee may also lead to the financing constraints of technological innovation enterprises. In the traditional financial market, representative financing channels such as banks generally require enterprises to provide collateral with strong realizable value, while innovative enterprises have a low proportion of tangible assets, weak mortgage ability, and low financing availability. For technological innovation activities, the lack of effective financial support may lead to the “flow of production” of a large number of innovative projects, which inhibits the improvement of regional innovation efficiency, and is ultimately not conducive to the optimization and upgrading of China's industrial structure and the establishment of an innovative country [5]. Digital finance, as a brand new form of financial industry, with its “inclusive” concept and “grassroots” characteristics, may be in line with the characteristics of financing needs and innovation environment of technology-innovative enterprises.

Recently, the academia and the industry put forward the “wisdom city” and the concept of “environmental protection” wisdom [6]. “Environmental wisdom” is the extension of the development of “digital green” and the deepening of the Internet and information technology in the field of environmental protection. On the basis of “digital environmental protection,” the “environmental protection wisdom” adds intelligent sensing system equipment in the front-end application, uses various information and communication technologies, and integrates the environment Internet of things through cloud computing, virtualization, and mainframe computers [7]. Building a new generation of network “smart” environmental protection systems integrating strong perception ability [8], intelligent processing ability, and comprehensive management ability provides more dynamic and accurate support for environmental management and decision-making, and digital environmental protection is the foundation of intelligent environmental protection. Compared with the traditional urban environmental governance mode, realizing the digitization and networking of environmental monitoring equipment is the basis of intelligent environmental protection. Although smart environmental protection and smart city construction are the inevitable trends of historical development, the practice of smart environmental protection in smart city construction is not plain sailing. Smart city construction brings both opportunities and challenges to the environmental protection industry. How to better realize the intelligent environmental protection in smart city is a major problem facing the world today. China, as a developing country actively advocating smart environmental protection and environmental protection city construction, should make efforts to find the reason.

## 2. Technology Trends

Big data has 3 V characteristics of variety [9], volume [10], and velocity [11]. Due to the integration and innovation of big data and different industries, the operation and service modes of traditional industries have changed, and new platforms, new models, and new business forms have been derived, such as Internet finance and car sharing. Finally, mass entrepreneurship and innovation is accelerating with the sharing and opening of big data. The digital economy is accelerated by technological innovation and technology-driven economic innovation. With the acceleration of big data technology and the integration of various sectors of the social economy, traditional industries can improve their productivity and innovation capacity and realize their digital transformation.

### 2.1. New Development Trend of Blockchain

The essence of blockchain is a distributed accounting synchronous updating ledger technology that collectively maintains a reliable database in a decentralized and trustless way. As the underlying technical support of Bitcoin, blockchain is essentially an imtamable distributed ledger, as well as a brand new distributed infrastructure and computing paradigm. Its basic ideas include using distributed networks to realize decentralized information processing, using consensus mechanism to establish trust between nodes, using asymmetric encryption and redundant distributed storage to realize information security, and using blockchain data structures to realize data information traceability.

In the era of digital economy, the development trends of blockchain are as follows: First, the virtual blockchain will be transformed into a real blockchain. Speculative currency speculation will cool, and blockchain's trust-building features will be taken seriously and applied to the real sector to promote the efficiency of the real economy. Second, cross-fusion. Blockchain will further accelerate the integration with new digital technologies such as big data, the Internet of things, and artificial intelligence. The development of blockchain technology and applications requires big data, the Internet of Things, artificial intelligence, and other next-generation information technologies as infrastructure support to expand the application space. Meanwhile, the development of blockchain technology and application plays an important role in promoting the development of the new generation of information technology industry [12]. Third, standards-led blockchain development will be more standardized. Blockchain in the industry has seen rapid development, but due to the differences in the industry, between users, the lack of uniform standards, the duplication, and waste of resources, in February 2018, China's ministry of industry of the chain block data format specification marked the blockchain technology standardization stage in essence.

Although the development and application of blockchain technology are relatively limited at present, the technology of blockchain is far from mature, and there are still many problems. However, with the increase in blockchain into future, chain blocks and the combination of the digital economy will increasingly close; the digital economy management platform based on blockchain is expected to become a public data sharing management infrastructure, and blockchain technology will gradually become the mainstream of the application; from the financial sector to the non-financial sector penetration, it will gradually become a new demand that subverts the traditional industry development.

### 2.2. New Development Trend of VR

VR is based on data acquisition, computer three-dimensional graphics technology, multimedia technology, interpersonal interaction technology, network transmission technology, three-dimensional display technology, and other technologies, all integrated to develop a new technology. As the digital economy continues to evolve, big data can provide granular support for immersive virtual scene, while virtual reality provides rich visualization solutions for big data. In this way, people's ability to analyze and process interactive big data is enhanced.

In the era of digital economy, the development of virtual reality technology has brought new industrial changes and business opportunities. Digital economy has driven the application and development of virtual reality in industrial design, virtual shopping, psychological therapy and rehabilitation, military simulation, and other fields. MIT Multimedia Experiment Center, Virtualitics, and other research institutions apply big data technology to VR scene construction to solve the problems that traditional 2D and 3D visualization systems are not capable of processing due to complex datasets, giving full play to the innate advantages of VR (immersion). The rollercoaster virtual space is based on NASDAQ data, allowing passengers to experience NASDAQ's rise and fall in the past 21 years from a first view. Master of Pie demonstrated how VR can be applied to big data analytics, where data are presented in a more natural and immersive way, allowing users to analyze and modify data in real time. According to Forbes, big data researchers using the technology can see four times as much information as a traditional computer screen “at a glance.”

### 2.3. New Trend of Sharing Economy Development

The rapid development of mobile internet has rapidly spawned a new business model based on big data, cloud computing, and third-party payment, namely the sharing economy. The essence of sharing economy is to eliminate sellers in the traditional sense, and it is digitalization that drives the progress of the elimination process. Digital technology makes it interact in the transaction process in the form of point-to-point connection, so as to improve the availability of services, reduce transaction costs, and enable consumers to enjoy the characteristics of productive services [13]. For example, in terms of shared travel, bike-sharing and car-sharing are developing rapidly. Didi Chuxing's operation data in 2017 show that in 2017, there were more than 20 billion route planning requests per day and more than 4500 TB of data were processed per day. Data analysis can help smart travel, achieve green travel, and improve urban planning. When it comes to housing, Airbnb has more than 120 million listings in more than 190 countries, and based on that data can accommodate an average of 400,000 people a night. The rapid development of sharing economy accelerates the growth of the digital economy. Based on the massive data generated by sharing economy, accurate matching is achieved through analysis and prediction, which accelerates the development of sharing economy. At the same time, based on the massive data generated by the sharing economy, the status quo and changing trend of urban transportation, employment, education and medical care, and other livelihoods can be interpreted, providing the decision-making basis for urban development. In the future, sharing economy will further expand its dimensions and service chain, carry out derivative services, promote more cross-border cooperation and innovation, and gradually spread to various industries, especially key fields such as education and medical care. At the same time, the sharing economy will gradually develop into the whole process, from consumption and production to distribution and circulation.

### 2.4. New Advancement Pattern of Internet of Things

With the vigorous development of the Internet of things, a variety of sensors and terminals can quickly access the network and gather together. At the same time, the number and structure of Internet devices have increased sharply at the same time, from PC to mobile phone, from tablet to the era of Internet of things. This development leads to the urgent need to measure unstructured information. It is assessed that there will be 50 billion associated detecting gadgets in 2020, producing 2.5 million terabytes of information each day, 2.38 times more than the ongoing Internet. The mix of the Internet of Things and the advanced economy has sped up its application in regions, for example, clinical observing frameworks, savvy home machine control, and operations and production network following. The fundamental advancement patterns of the Internet of Things in the computerized economy time are as per the following: First, sensor innovation is creating towards high accuracy to advance all over information assortment and transmission. The fame of wearable gadgets advances the portability of the Internet of Things, and high-accuracy sensor innovation works on the awareness and precision of observing. Second, it can combine with savvy gadgets to advance the mental prowess of the Internet of things. During the time spent on savvy gadget control, the observing information of shrewd watches/wristbands in wearable gadgets can be sent to the medical clinic progressively to understand the ongoing checking administration of the client's body and stay away from the event of related illnesses. Third, the Internet of Things' biological system has turned into the principal type of utilization landing. IT goliaths have additionally organized the IoT biological system in a steady progression. For instance, Apple has framed a multi-stage IoT environment including shrewd home HomeKit, wearable gadget HealthKit, and vehicle IoT CarPlay. Google proposed Project IoT and delivered the Brillo IoT fundamental working framework. Huawei has delivered Lite OS, a lightweight Internet of Things working framework, and NB-IoT, a start to finish answer for constructing an Ocean Connect environment.

### 2.5. New Patterns in AI Advancement

With the collection of computerized assets, the improvement of processing power, and the improvement of organization offices, the flood of huge information has turned profound gaining and man-made brainpower from a fantasy into the real world, and man-made reasoning is entering another phase of cross-line combination, with profound application and driving turn of events. In the field of biometric acknowledgment, the FACE dataset (NGI) developed by the Federal Bureau of Investigation (FBI) has gathered 117 million American grown-ups' fingerprints, iris, face, and other biometric information. Face acknowledgment innovation can be utilized to figure out the objective through photographs. In the clinical field, man-made reasoning innovation can be utilized to handle the gigantic information and data gathered to figure out the pertinent obsessive premise and important cases, and work on the precision of conclusion and navigation. Then, the innovation of computer economy and human consciousness will be more focused on deep learning and artificial intelligence, key innovation. Accelerate the application of computer reasoning in currency, clinical and program driven, and turn it into common sense, thus promoting a new round of modern transformation.

## 3. Technological Cross and Integration in the Era of Digital Economy

Digital economy is most rapidly developing in modern times; innovation is the most active and most widely emerging economic activity; its core elements are the data resources, the key technology of data mining, and utilization of resources; its essence is the large data, cloud computing, Internet of things, artificial intelligence, and blockchain: five new digital technologies leading the digital transformation.

Big data technology promotes the sharing economy enterprise's innovation and development, but has many problems, such as information security, privacy, and poor regulation; relying only on big data sharing technology has made it unable to maintain the innovation of new economic models, and blockchain technology has encryption sharing; distributed books do not tamper with the advantages. It provides new technical support for the circulation and sharing of data and can be complementary with big data technology. Blockchain technology in the era of big data has three characteristics: First, the mass storage of big data and distributed computing technology improve the value and use space of blockchain data. With its reliability, security, and imtamability, blockchain provides a strong guarantee for the open sharing of big data under the premise of privacy protection, freeing more big data. Second, blockchain has traceability features, which can effectively improve data quality. Blockchain can record every step of data processing in detail, including data collection, transaction, circulation, and computational analysis, such that the quality of data has a strong trust endorsement. Third, blockchain can standardize the use of data and fine-tune the scope of authorization. Data trading and circulation after desensitization can prevent the formation of information islands and promote the gradual formation of globalized data trading scenarios; the effective combination of digital economy with blockchain and Internet of Things will also lead a new round of economic revolution [14, 15].

### 3.1. The Integration of New Digital Technologies Promotes the Innovative Development of the Digital Economy

Digital economy is most rapidly developing in modern times; innovation is the most active and most widely emerging economic activity, and its core elements are the data resources, the key technology of data mining, and utilization of resources; its essence is the large data, cloud computing, network, artificial intelligence, and blockchain—five new technologies leading to the digital transformation of the economy. New digital technologies have profoundly changed the way of thinking, production, and the life of mankind, making economic digitalization an important driving force for innovative economic development.

## 4. Application Innovation Trend in the Digital Economy Era

“Tmall International,” with more than 40 million service users, accounted for half of the online shopping market in China. In this retail ecosystem, relying on the Internet and big data, Tmall International relies on Alibaba's powerful data ecosystem to help a large number of overseas merchants to break through the brand online and offline system and establish a global supply chain. Brand operators, such as Australian natural health brand Swisse, share data with Alibaba to predict consumer buying trends and potential demand [16].  Figure 1 shows the new retail applications in the digital economy era.

The fresh market of new retail has become a trillion-level market, and each giant has taken the lead. “Hema Xiansheng” is a typical representative. It uses digital technology and comprehensive performance links in the supply chain, sales, and logistics to achieve full digital, intelligent, optimized workflow, reduce ineffective work, to shop for their goods, shelves, picking, packing, distribution and other tasks, homework personnel and assignments, which can be identified by intelligent devices; the error rate is extremely low, and the whole system is divided into foreground and background. Users place orders within 10 minutes of sorting and packaging, and it takes 20 minutes to achieve delivery within 3 km.

### 4.1. Digital New Technology Leads to Production and Manufacturing to Realize Intelligent Production

The IoT combines artificial intelligence, cloud computing, and big data analytics to analyze the collected data through a large number of connected sensors that can monitor complex physical and mechanical performance in real time to optimize production and perform proactive maintenance, improving efficiency and generating information that can be used to develop new processes. The data collected can also be used to analyze other relevant areas beyond manufacturing, such as reducing energy consumption and network resource investment. In product production planning and process control, the factory in the production process using smart devices and sensors to collect the production process to produce large amounts of data, dig into these data and applications, and optimize processing methods, processing sequence, and system technology indexes such as cutting parameters, the real-time monitoring of production process, troubleshooting, and feedback adjustment.

### 4.2. Digital New Technology Leads to Operation Optimization and Achieves Lean Management

The production process, equipment working conditions, process parameters, and other information can be collected in real time through the Internet of things, and product quality and defects can be detected and counted. In the offline state, machine learning technology is used to mine the relationship between product defects and the historical data of the Internet of Things and form control rules. In the online state, through enhanced learning technology and real-time feedback, it can control the production process to reduce product defects. At the same time, it can integrate expert experience to continuously improve learning results. In the maintenance service link, the system uses sensors to monitor the status of the equipment and establishes an analysis model of the equipment failure through machine learning. Before the failure occurs, the workpiece that may fail is replaced, so as to ensure the continuous trouble-free operation of the equipment. In terms of supply chain management and optimization, enterprises can use geographic big data analysis technology to integrate and optimize supply chain distribution networks, optimize purchase time, purchase quantity, warehouse allocation, etc., to improve inventory efficiency. In the field management optimization, artificial intelligence can also be used in digital field equipment life cycle health management, machine vision-based field safety, field environmental management, etc.

### 4.3. New Trend of Smart City Application

The wisdom of the city's development is inseparable from the urban informatization infrastructure construction; infrastructure to collect and record large data resources for professional analysis and management decision support is needed; blocking the use of chain technology to a certain extent can solve urban problems such as data storage and safety. McKinsey predicted in a research report based on western industry data that the application of big data would save more than 100 billion euros in operating costs for the governments of European developed countries and make the Medical insurance of the United States health sector costs reduce by 8 percent, saving more than US $300 billion annually.

#### 4.3.1. The Scientific Development of the Urban Economic Structure, Spatial Structure, and Social Structure Will Be Realized by Digital New Technology

Specifically, in urban planning, big data, as an important strategic asset, is conducive to the cultivation of a new concept of urban planning combining “top-down” and “bottom-up” approaches, and can promote the realization of a new trend of integrating GIS-based urban planning system into urban planning. Innovative data acquisition and processing technologies, on-site research methods, new methods of programming, public participation in planning, and new methods of urban planning will eventually make smart city planning reach a new height and form a progressive smart city planning system.

#### 4.3.2. Digital New Technology Can Achieve Accurate Management of Urban Social Order, Ecological Environment, and Infrastructure

The intelligent perception and recognition technology of artificial intelligence can be used to collect and coordinate urban traffic, logistics, energy, environment, and other information in real time. According to the data-driven formation of urban decision-making mechanism, digital intelligent management of the city finally realize the intelligent allocation of public resources. Using artificial intelligence technology, it can automatically digest the unstructured massive surveillance video data generated by the security industry that cannot be calculated statistically. At present, artificial intelligence has penetrated into every industry and department to varying degrees. By collecting data in various fields, it can make intelligent analysis and effectively use urban information, enhance the efficiency of urban management, save resources, protect the environment, provide decision support for sustainable development, and promote the construction of smart cities.

### 4.4. New Trends in Mobile Medical Applications

#### 4.4.1. Digital New Technology Helps Chronic Disease Prevention and Health Management

Based on the Internet of things, a national public health monitoring platform will be built. Health departments can strengthen continuous medical observation, timely discover potential disease risks, and give early warning and prevent chronic diseases and epidemics through the electronic medical record database covering the whole country. In addition, patients' personal data, electronic medical records, and ethnic database in China can also be used to quickly detect diseases and identify the causes [17], so as to build personalized rehabilitation treatment programs suitable for Chinese people. In the field of practice, “Shuangquan (comprehensive screening and whole-process management) Plan” and Google's “Global Influenza Map” are important manifestations of big data in the management of mass prevention and treatment of chronic diseases and the prediction of high incidence areas. Finally, by combining the Internet of Things with blockchain, all kinds of medical equipment and services can be connected to monitor residents' and patients' exercise and health data, and obtain fitness, medical, physical, and exercise monitoring data. The anonymity of blockchain ensures patients' privacy. At the same time, it can get through the information channel between hospitals, financial insurance, pharmaceutical factories, and other relevant departments.

#### 4.4.2. New Digital Technologies to Assist Clinical Decision-Making

Artificial intelligence technology is used to analyze diverse, multi-source, fragmented, and unstructured medical data, and to support clinical decision-making through a series of means such as etiology identification, clinical data comparison, clinical decision support, and remote patient data analysis, so as to achieve precision medicine. In terms of clinical data comparison, the best treatment approach can be obtained by matching the medication status of patients with the same type. In clinical decision support, deep learning and other methods are applied on medical datasets to realize intelligent diagnosis and treatment.

#### 4.4.3. Digital New Technology to Assist Medical Research and Development

Big data can be integrated into every stage of medical research and development, play a key role in every link of research and development, and can liberate the pharmaceutical research and development industry from the dilemma of high investment, high risk, and long cycle. Through data summary and analysis, the influence of big data on the whole process of drug R&D can be reflected in three stages: In the stage of drug project approval, we used big data to find drugs urgently needed in the market, quickly analyzed pre-clinical trials of drugs, identif effective target drugs, and analyzed technology to process drug data (for example, there are nearly 30 diabetes drugs in the market around the world, and each drug has about 20,000 pages of literature). In the stage of drug development, chemical structure big data can be used to quickly establish chemical structures or carry out targeted structural transformation, compare pharmaceutical processes, and optimize pharmaceutical processes. In the stage of clinical trials, big data of clinical trials can be used to establish pharmacodynamic models, evaluate efficacy, predict adverse reactions, and speed up clinical trials.

### 4.5. New Trend of Personalized Education Application

The new digital technology is the scientific power to promote the innovation and development of education. Educational big data is a collection of all the data generated in the whole process of educational activities and collected according to the needs of education for educational development and can create huge potential value. Driven by big data in education, new digital technologies such as blockchain and artificial intelligence are becoming a subversive force to promote innovation and reform the education system. Compared with traditional education, the realization of personalized education application depends on the application of new digital technology in the following aspects.

#### 4.5.1. New Digital Technologies Help Learners Discover and Develop Their Potential and Improve Their Academic Performance

Artificial intelligence and learning science are combined to form a new field, Educational Artificial Intelligence (EAI). At present, a large number of educational AI systems have been applied in schools. These systems integrate educational AI and educational data mining (EDM) technologies (such as machine learning algorithms) to track students' behavioral data and predict their learning performance to support personalized learning. Through artificial intelligence, “teaching, learning, and evaluation” can be organically combined. Schools and other institutions can automatically mark learning materials through NLPs and other artificial intelligence technologies to evaluate students' knowledge points, realize real-time feedback and accurate review, and realize collaborative supervision and self-supervision to promote learning. For example, the American KHAN system can clearly see students' learning progress, knowledge mastery, and teacher's recommendation.

#### 4.5.2. Digital New Technology Helps Teachers Determine the Most Effective Teaching Method and Optimize the Teaching Process

Big data matching algorithm helps to realize learning recommendation, analyze learning data and course data, and can also be used to realize adaptive learning. For example, Knewton company of the United States has used big data to provide digital course materials, which has realized dynamic and continuous adaptation to the unique needs of each student. As Internet technology continues to penetrate into the education industry, big data behavior analysis means are constantly promoting traditional education from statistical analysis for groups to behavior analysis for individuals. After acquiring big data, on the one hand, intelligent means, such as association analysis and recommendation algorithm, can be used to customize personalized teaching contents and methods, automatically discover rules and use them for prediction. For example, “Xuetang Online” can dig into the value of MOOC and adjust courses accordingly. On the other hand, according to online and offline data analysis, it can timely guide students to solve problems. Real-time feedback of learning data is beneficial to explore students' interests and characteristics, so as to realize the exchange of online and offline data, realize supervised learning, judge the degree of knowledge mastery of students, and timely modify teaching ideas and methods.

The new digital technology helps realize the mode of two-way education delivery. Using virtual reality technology, teaching content can be organized according to their own ideas and knowledge structure can be constructed, and this organization information is not a simple linear structure. Virtual reality technology connects these complicated knowledge into a network, providing students with a vivid knowledge structure. It includes not only the basic content of the subject, but also the logical relationship between the contents of the subject. It pays attention to both the formation process of knowledge and the structure of knowledge. Through the coordination of our vision, hearing, and touch, the unity and flexibility of the teaching content can be perfectly combined. For many abstract concepts and things, virtual reality can be restored to real scenes, allowing students to try different experiments, or even simulate micro scenes, to explore the essence of things or phenomena, without worrying about any danger.

### 4.6. New Trend of Region-Wide Tourism Application

With the arrival of the era of mass tourism, the new digital technology is playing an increasingly important role in the tourism industry. The development of region-wide tourism no longer depends on perceptual experience, but needs to rely on new digital technologies to make decisions.

1. LBS, search engine, online travel agency (OTA), and other tourism data can help the tourism industry's market segmentation and positioning. Specifically, the tourism climate index can be used to predict the future growth of the tourism market. Through the analysis of tourists' preference, the tourism market is segmented. Through the analysis of tourist source, one can judge the distribution of main tourist source markets. Through the analysis of potential markets, we can explore the depression of regional tourism markets and through the analysis of the loss of tourists, we can improve the tourism market conversion rate.
2. Based on the Internet of Things technology and cloud computing platform, we can integrate various tourism-related businesses and professional resources, acquire big data, analyze, integrate, and share the obtained data accurately, and provide strong support for tourism managers to make decisions and meet the personalized needs of tourists. For example, the construction of user portraits, personalized tourism strategy recommendation, innovation of traditional tourism department's organizational forms, including personalized recommendation matching destinations, tourist attractions and routes, personalized recommendation of hotels and locations, personalized recommendation of direct flight or transfer, and personalized recommendation of popular food and shopping sites can be achieved. TripAdvisor has done well in this area. As the world's leading travel planning and booking site, it catalogues more than 500 million reviews and recommendations from travelers around the world, covering 7 million homes, restaurants, and attractions in more than 190 countries.
3. Based on weather, hotel, traffic, and other data, one can realize the number of tourists forecast and safety warning. Deeply analyze the daily, weekly, seasonal, and holiday traffic characteristics of the scenic spot, as well as the impact of weather, traffic, and historical traffic data on the scenic spot, and then control the distribution of tourists in the scenic spot in real time according to the scenic spot forecast and legal holiday traffic, so as to effectively prevent tourists from crowding and stampede in the scenic spot.

## 5. Conclusion

Based on the perspective of digital finance and technological innovation, this paper analyzes its application in economic development, green economy, and sustainable development. With the continuous development of technological economy, methods such as artificial intelligence, Internet of Things, big data, and cloud computing become increasingly mature. Economic development is inseparable from the empowerment of technology. At present, China is still facing various difficulties and problems in economic development and application, and hence we should make full use of the information advantages of new digital technology, form subversive technological change, and expand the application of advanced technology in depth, so as to promote the development of the digital economy.

## Figures and Tables

**Figure 1:** New retail applications in the digital economy era.

## Data Availability

The experimental data used to support the findings of this study are available from the corresponding author upon request.

## References

[1] Schumpter J. A. (1942). *Captitalism, Socialllism and Democracy*.

[2] Nanda R., Nicholas T. (2014). Did bank distress stifle innovation during the great depression?. *Journal of Financial Economics*.

[3] Guo F., Kong S. T., Wang J. (2016). General patterns and regional disparity of internet finance development in China: evidence from the peking university internet finance development index. *China Economic Journal*.

[4] Stiglitz J. E., Weiss A. (1981). Credit rationing in markets with rationing credit information imperfect. *American Economic Review*.

[5] Aghion P., Fally T., Scarpetta S. (2007). Credit constraints as a barrier to the entry and post—entry growth of firms. *Economic Policy*.

[6] Atiquzzaman M., Yen N., Xu Z. Big data analytics for cyber-physical system in smart city2021.

[7] Cheng Y., Meng H., Yuan L., Lei Y. Research on edge computing technology of internet of things based on intelligent and environmental protection.

[8] Yang Q. (2019). The smart city of Changsha, China—sciencedirect. *Smart City Emergence*.

[9] Einav L., Levin J. (2014). Economics in the age of big data. *Science*.

[10] Lynch C. (2008). Big data: how do your data grow?. *Nature*.

[11] Lazer D., Kennedy R., King G., Vespignani A. (2014). The parable of google flu: traps in big data analysis. *Science*.

[12] Li J., Peng Z., Liu A., He L., Zhang Y. Analysis and future challenge of blockchain in civil aviation application.

[13] Schor J., Fitzmaurice C. (2015). Collaborating and connecting: the emergence of the sharing economy. *Handbook on Research on Sustainable Consumption*.

[14] Zhou Y., Wang K., Liu H. (2018). An elevator monitoring system based on the internet of things. *Procedia Computer Science*.

[15] Liu R., Yang B., Zio E., Chen X. (2018). Artificial intelligence for fault diagnosis of rotating machinery: a review. *Mechanical Systems and Signal Processing*.

[16] Umair A., Hui P., Muhammad K., Yan C., Akram Z. (2018). Factors affecting online impulse buying: evidence from Chinese social commerce environment. *Sustainability*.

[17] Zhang J., Hu J., Huang L., Zhang Z., Ma Y. (2016). A portable farmland information collection system with multiple sensors. *Sensors*.

